# The Aminopyridinol Derivative BJ-1201 Protects Murine Hippocampal Cells against Glutamate-Induced Neurotoxicity via Heme Oxygenase-1

This article has been retracted.

**DOI:** 10.3390/molecules21050594

**Published:** 2016-05-05

**Authors:** Dong-Sung Lee, Tae-Gyu Nam, Byeong-Seon Jeong, Gil-Saeng Jeong

**Affiliations:** 1 College of Pharmacy, Chosun University, Dong-gu, Gwangju 61452, Korea; dslee2771@chosun.ac.kr; 2 Department of Pharmacy, Hanyang University, Ansan 15588, Korea; tnam@hanyang.ac.kr; 3 College of Pharmacy, Yeungnam University, Gyeongsan 38541, Korea; 4 College of Pharmacy, Keimyung University, Daegu 42601, Korea

**Keywords:** aminopyridinol compound BJ-1201, neuroprotection, aminopyridinol HT22, heme oxygenase-1, nuclear transcription factor erythroid-2 related factor 2

## Abstract

Glutamate is the major excitatory neurotransmitter in the brain. It can cause neuronal cell damage in the context of oxidative stress. BJ-1201 is a derivative of the compound aminopyridinol, which is known for its antioxidant activity. In this study, we examined the effect of BJ-1201, a 6-(diphenylamino)-2,4,5-trimethylpyridin-3-ol compound, on neuroprotection in HT22 cells. Our data showed that BJ-1201 can protect HT22 cells against glutamate-induced cell cytotoxicity. In addition, BJ-1201 upregulated heme oxygenase-1 (HO-1) to levels comparable to those of the CoPP-treated group. BJ-1201 treatment induced phosphorylation of JNK, but not p38-MAPK or ERK. It also increased the signal in the reporter assay based on β-galactosidase activity driven by the nuclear transcription factor erythroid-2 related factor 2 (Nrf2) promoter harboring antioxidant response elements (AREs) and induced the translocation of Nrf2. These results demonstrate that BJ-1201 may be a good therapeutic platform against neurodegenerative diseases induced by oxidative stress.

## 1. Introduction

Oxidative stress is involved in several neurodegenerative diseases, such as Alzheimer’s disease (AD), Huntington’s disease (HD) and Parkinson’s disease (PD) [1]. In particular, production of reactive oxygen species (ROS) followed by subsequent oxidative modification of biomolecules, such as proteins, DNA and lipids, has been implicated in the pathological events of neurodegenerative diseases [2]. Glutamate is the major excitatory neurotransmitter in the brain and can cause neuronal cell damage in conjunction with oxidative stress. Glutamate toxicity also has been shown to induce neuronal cell death through both receptor-initiated excitotoxicity and non-receptor-mediated oxidative stress. Immortalized neuronal HT22 cells, originating from mouse hippocampus, lack functional ionotropic glutamate receptors, thus HT22 cell is damaged by glutamate via the non-receptor-mediated oxidative pathway [3]. It has also been widely used to identify substances with protective effects against oxidative stress in brain cells [4,5].

Antioxidant enzymes, such as thioredoxin reductase, glutathione peroxidase, catalase and heme oxygenase-1 (HO-1), exist in our body as a cellular defense mechanism against oxidative stress [6,7]. HO-1 catalyzes the oxygen-dependent degradation of heme to biliverdin, iron, and carbon monoxide using reducing equivalents such as NADPH [8]. Therefore, HO-1 regulates homeostasis of pro-oxidative heme iron. Previous reports have suggested that its expression protects HT22 cells from glutamate toxicity [9]. HO-1 is included in the family of antioxidant response element (ARE)-containing genes and its expression is regulated by nuclear transcription factor erythroid-2 related factor 2 (Nrf2) [10]. Nrf2 is a master regulator of detoxifying/antioxidant phase II enzymes, including HO-1. Nrf2 binds to a specific DNA sequence (ARE) within the promoter region of phase II enzymes to enhance their transcription. HO-1 gene expression is induced by stress-associated stimuli such as inflammation, UV light and hypoxia whose signals are mediated through mitogen-activated protein kinases (MAPKs) activation or by non-stressful stimuli such as c-GMP and c-AMP. Although the physiological role of HO-1 in oxidative stress is not fully understood, due to its function in cytoprotection in stressed environments, its induction is generally considered to be a cellular defense mechanism. Recently, many studies have reported that small molecules, such as geniposide [11], sulfuretin [12], butein [13], and puerarin [14] have inhibitory effects on oxidative stress-induced neuronal damage through the induction of HO-1. Thus HO-1 inducers with no implication of cellular stresses may have potential therapeutic values. BJ-1201 is a derivative of the compound aminopyridinol, which is known for its antioxidant activity [15]. It was tested elsewhere for antiangiogenic activity, only displaying very mediocre activity [16]. In this study, we investigated the antioxidant activity of BJ-1201 from a different perspective and here report that this compound has protective activity against oxidative stress in HT22 cells.

## 2. Results

### 2.1. BJ-1201 Inhibits Glutamate-Induced Oxidative Neurotoxicity

To determine the effect of BJ-1201 on glutamate-induced cell death by MTT assay, HT22 cells were pretreated with different concentrations of BJ-1201 (up to 20 μM). 1–20 μM BJ-1201 did not affect the cells significantly, suggesting that these concentrations were non-toxic to HT22 cells (Figure 1b). In addition, we have already evaluated the toxicity effects of glutamate (0, 0.5, 2, 5, 10, 20 mM) on cell viability in HT22 cells. Glutamate was shown to significantly reduce cell viability to 65.8% ± 1.3% at 5 mM and 42.2% ± 3.2% at 10 mM for 12 h compared to that of the untreated cells (Data not shown). In addition, we have also checked the glutamate-induced ROS production to 149.35% ± 6.9% at 5 mM and 208.77% ± 8.3% at 10 mM for 12 h (data not shown). Therefore, in our study, glutamate was used at concentrations of 10 mM, respectively. Next, we wanted to evaluate the cytoprotective effects of BJ-1201 on glutamate-induced cytotoxicity in HT22 cells. Treatment with 10 mM glutamate for 12 h increased HT22 cell death up to 35% compared to untreated cells (Figure 1c). On the other hand, treatment with BJ-1201 increased the cell viability of glutamate-treated cells in a dose-dependent manner. Glutamate also induced ROS generation in HT22 cells as determined from the fluorescent signal (Figure 1d). As shown in Figure 1d, BJ-1201 effectively decreased ROS production that was induced by glutamate treatment. Trolox, a water-soluble derivative of α-tocopherol, was used as a positive control. These results showed that BJ-1201 has cytoprotective and ROS-scavenging effects in hippocampal HT22 cells.

### 2.2. BJ-1201 Upregulates HO-1 Expression

To determine the relationship between BJ-1201 and HO-1 protein expression in HT22 cells, we incubated the cells for 18 h in the presence of BJ-1201 at the indicated concentrations. BJ-1201 increased HO-1 expression in HT22 (Figure 2a) in a dose-dependent manner. Cobalt protoporphyrin IX (CoPP), a well-known HO-1 inducer, was used as a positive control (10 μM).

In line with the increase in protein expression of HO-1 by BJ-1201, BJ-1201 treated cells showed higher enzymatic activity of HO in a dose-dependent manner (Figure 2b). These results demonstrate that BJ-1201 directly affects HO-1 protein levels.

### 2.3. BJ-1201 Activates MAPK in HT22 Cells

MAPK’s are activated in response to oxidative stress and other forms of external stress. Several studies showed that the activation of the MAPK pathway can induce HO-1 expression *in vitro* [17,18,19]. Since BJ-1201 increased the expression level of HO-1, we wanted to examine the effect of BJ-1201on the activation of MAPK’s in HT22 cells to further investigate the relationship between BJ-1201-induced HO-1 expression and MAPK activation. We incubated the cells with 20 μM BJ-1201 for 0–60 min, and then evaluated MAPK expression. As shown in Figure 3b, phosphorylation of JNK was activated by BJ-1201 in HT22 cells, whereas phosphorylation of ERK and p38 was unaffected by BJ-1201 (Figure 3).

### 2.4. Involvement of JNK in BJ-1201-Inducing HO-1 Expression and Glutamate-Induced Neurotoxicity

We determined the effects of specific MAPK inhibitors on HO-1 protein expression induced by BJ-1201 (Figure 4). Cells were incubated with BJ-1201 (20 μM) in the presence and absence of JNK inhibitor (SP600125), ERK inhibitor (PD98059) or p38 MAPK inhibitor (SB203580). Inhibition of JNK pathway significantly inhibited BJ-1201-induced HO-1 expression whereas the inhibition of either ERK or p38 MAPK pathway did not affect BJ-1201-induced HO-1 expression (Figure 4a). Further evidence of HO-1 induction via the JNK pathway was provided by the fact that the inhibitor did not induce HO-1 expression (Figure 4a). Thus, while the inhibition of ERK or p38 MAPK pathway did not affect BJ-1201-induced viability, inhibition of the JNK pathway reversed the viability obtained in the presence of BJ-1201, resulting in the same viability as glutamate alone (Figure 4b). Taken together, these results suggested that BJ-1201 increased HO-1 expression through JNK phosphorylation in HT22 cells. In addition, we also examined whether BJ-1201-induced HO-1 induction mediated these protective action. HT22 cells were co-treated with the absence or presence of BJ-1201 or SnPP. SnPP significantly inhibited the BJ-1201-mediated cytoprotection (Figure 4b).

### 2.5. BJ-1201 Induced Upregulation and Nrf-2 Nuclear Translocation in HT22 Cells

We examined whether BJ-1201 induced nuclear translocation of Nrf2 in HT22 cells (Figure 5a,b). The cells were treated with BJ-1201 (20 μM) for 0.5, 1, or 1.5 h. Nrf2 levels in the cytosolic fraction decreased in response to treatment.

In contrast, Nrf2 levels in the nuclear fraction increased significantly upon treatment with BJ-1201, demonstrating translocation of Nrf2, which plays an important role in the transcriptional activation of HO-1 gene [18,19]. We further investigated ARE-activation by BJ-1201 using luciferase assays. Figure 5 showed that BJ-1201 dose-dependently increased ARE-luciferase activity.

## 3. Discussion

In our previous studies, we have been investigated the synthesis of aminopyridinol compounds, including BJ-1201, a 6-(diphenylamino)-2,4,5-trimethylpyridin-3-ol derivative. In addition, the aminopyridinol derivatives were tested elsewhere for antiangiogenic activity, only resulting in very mediocre activity [15,16]. BJ-1201 is already well known for its antioxidant activity, however, there have been no studies on the molecular targets of aminopyridinol derivatives including BJ-1201 and the mechanisms underlying their anti-neurodegenerative biological activities. Therefore, the present study focused on the molecular targets and specific mechanisms underlying the anti-neurodegenerative activities of BJ-1201. In this study, we investigated the effect of BJ-1201 on neuroprotection in HT22 cells. We first investigated the protective effects of BJ-1201 against glutamate-induced cytotoxicity in HT22 cells. The results showed that 12 h-pretreatment with BJ-1201 (1–20 μM) dose dependently inhibited glutamate-induced cell death, and also effectively suppressed glutamate-induced reactive oxygen species (ROS) generation (Figure 1). Furthermore, the data revealed the induction of HO-1 and HO-1 activity by BJ-1201 in HT22 cells (Figure 2). Additionally, by using HO-1 inhibitor, SnPP, we showed that BJ-1201 affected HO-1 induction (Figure 4). The induction of HO-1 expression is required to suppress glutamate-induced reactive oxygen species generation. These results suggested that the cytoprotective effects of BJ-1201 might be due to the induction of HO-1.

Oxidative stress via excess ROS plays an important role in cell dysfunction and the initiation and progression of many neurodegenerative diseases such as Alzheimer’s disease, Parkinson’s disease, neuronal stroke, carcinogenesis, and ischemia [20,21]. Glutamate is a neurotransmitter in the central nervous system. In HT22 cells, glutamate also induces oxidative stress and increases ROS production. ROS-scavenging activity, which is related to oxidative stress of candidate substances, is a suitable indicator of potential antioxidant effects. The hippocampal cell line (HT22), [22,23] a neuronal line derived from mouse hippocampus, is one of the cell lines used frequently in such experiments. HT22 cells have been used as an *in vitro* model for studying the mechanism of oxidative glutamate toxicity. Glutamate is the main excitatory neurotransmitter in the central nervous system (CNS). Glutamate toxicity has been shown to induce neuronal cell death through both receptor-initiated excitotoxicity and non-receptor-mediated oxidative stress [24,25]. Glutamate induces oxidative stress by inhibiting the cellular uptake of cystine via the cystine/glutamate transport system, Xc^−^, leading to depletion of glutathione, increased ROS production, and elevated Ca^2+^ levels [26,27]. This immortalized neuronal HT22 cells, originating from mouse hippocampus, lacks functional ionotropic glutamate receptors, thus excluding excitotoxicity as a cause for glutamate triggered cell death [3,28]. On the other hand, there are several recently publications demonstrating that the expression of NMDA receptor, a major contributor of glutamate-induced excitotoxicity, is very low in undifferentiated HT22 cells [29,30]. The system Xc-cystine/glutamate exchanger present in the astrocytes releases glutamate from the astrocytes to extracellular compartment to over-stimulate the extrasynaptic NMDA receptors in neurons. This in turn contributes to excitotoxic neuronal loss in ischemic stroke [29,30]. In this study, we provided evidence to support the view on the neuroprotexctive effects of BJ-1201 via up-regulation of HO-1 expression in glutamate-induced oxidative HT22 cells damage.

HO-1 is the rate-limiting enzyme in heme catabolism under the conditions discussed above. It is induced in a number of cell types by a range of stimuli, including LPS, proinflammatory cytokines, heavy metals, UV light, heat shock, and hypoxia [1,31]. HO-1 catalyzes the degradation of heme, producing iron, carbon monoxide, and biliverdin [7]. Biliverdin is subsequently converted to bilirubin, a powerful antioxidant, by biliverdin reductase [32]. We used SnPP, an inhibitor of HO-1, to confirm that the protective effects of BJ-1201 were due to HO-1 signaling (Figure 4). The neuroprotective effects of BJ-1201 may occur through HO-1 signaling pathways.

Previous studies have shown that several small molecules can modulate the activity of MAPKs in several cell lines, including HT22 cells. Next, we examined whether BJ-1201 effected MAPK pathway activation. BJ-1201 activated JNK phosphorylation in HT22 cells (Figure 3b). The efficacy of the MAPK inhibitors was evaluated by analyzing their effects on the phosphorylation of p38, JNK and ERK (Figure 3). Additionally, evidence has shown that MAPK regulates the nuclear translocation of Nrf2. Nrf2 is a transcription factor. Its regulation of oxidative stress and its signal transduction pathway include HO-1. When stimulated by inducers, Nrf2 is released from keap1 and translocates to the nucleus [33]. It dimerizes with other cofactors and binds ARE [34]. We investigated the potential involvement of BJ-1201 in the nuclear translocation of Nrf2, which has been shown to be important in ARE-induced gene induction of phase II detoxification enzymes and antioxidant proteins, in response to a number of stimuli, including laminar flow, oxidative stress, and chemopreventive agents, it also regulates oxidative stress-induced HO-1 expression in murine peritoneal macrophages [35,36,37]. Nrf2 is among antioxidant activities elicited by BJ-1201 (Figure 5a). Moreover BJ-1201 increased ARE-luciferase activity in a dose-dependent manner (Figure 5b). MAPK and Nrf2 are part of the neuroprotective signaling cascades that also regulate HO-1 expression in mouse hippocampal cells. A previous study demonstrated that HO-1 blocked neutrophil trafficking in acute damage by suppressing neutrophil rolling, adhesion and migration, suggesting that the HO-1 pathway may regulate neuroprotective action. Similarly, our data showed that BJ-1201 increased HO-1 expression and activity in a dose-dependent manner. Figure 5 clearly demonstrated a decisive role for HO-1 enzymatic activity in the neuroprotective effects exerted by BJ-1201.

## 4. Materials and Methods

### 4.1. Materials

Dulbecco’s modified Eagle’s medium (DMEM), fetal bovine serum (FBS), antibiotics and other tissue culture reagents were purchased from Gibco BRL Co. (Gaithersburg, MD, USA). Lipopolysaccharide (LPS), 6-hydroxy-2,5,7,8-tetramethylchroman-2-carboxylic acid (Trolox), and 3-(4,5-dimethylthiazol-2-yl)-2,5-diphenyltetrazolium bromide (MTT) were purchased from Sigma Chemical Co. (Sigma-Aldrich, St. Louis, MO, USA). Cobalt protoporphyrin IX (CoPP), Tin protoporphyrin IX (SnPP), PD98059, SB203580 and SP600125 were purchased from Enzo (Enzo Lifesciences, Farmingdale, NY, USA). Primary antibodies, including Heme oxygenase-1 (HO-1) and Nuclear transcription factor erythroid-2 related factor 2 (Nrf2) antibodies, were purchased from Abcam (Abcam Plc, Cambridge, UK). Phosphorylated extracellular signal-regulated kinase 1/2 (p-ERK), phosphorylated JNK (p-JNK), and phosphorylated p38 (p–p38) antibodies and secondary antibodies used for western blot were purchased from Cell Signaling Technology (Cell Signaling Technology Inc., Beverly, MA, USA). All other chemicals were obtained from Sigma Chemical Co. BJ-1201, as a derivative of the aminopyridinol compound, was obtained from Dr. Jeong at Yeungnam University as previously described [16].

### 4.2. Cell Culture

Mouse hippocampal HT22 cells were obtained from Dr. In Hee Mook at Seoul National University (Seoul, Korea). The culture medium used in the experiments was Dulbecco’s modified Eagle’s medium (Gibco-BRL) and minimum essential medium Eagle (MEM) alpha containing 10% fetal bovine serum (Gibco, Cat. 16000-044) and 1% Antibiotic-Antimycotic (Gibco, Cat. 15240). The cells were maintained at 37 °C in a humidified atmosphere containing 5% CO_2_. Each cell line was subcultured every 2 or 3 days.

### 4.3. Cell Viability

Cell viability was determined by the 3-(4,5-dimethylthiazol-2-yl)-2,5-diphenyltetrazolium bromide (MTT) assay. The cells were plated in 96-well plates at a density of 1 × 10^4^ cells/well. After culturing, MTT reagent (5 mg/mL) was added to each well and incubated for 4 h, the supernatants were discarded, and the cells were dissolved in dimethyl sulfoxide (DMSO). The absorption was measured at 590 nm using a microplate reader (Molecular Devices, Sunnyvale, CA, USA).

### 4.4. Measurement of Reactive Oxygen Species

For the measurement of reactive oxygen species, HT22 cells (2.5 × 10^4^ cells/mL in 24-well plates) were treated with 10 mM glutamate in the presence or absence of BJ-1103 and incubated for 12 h. After washing with PBS, the cells were stained with 10 μM 2′,7′-dichlorofluorescein diacetate (DCFDA) in Hanks’ balanced salt solution for 30 min in the dark. The cells were then washed twice with PBS and extracted with 1% Triton X-100 in PBS for 10 min at 37 °C. Fluorescence was recorded with an excitation wavelength of 490 nm and an emission wavelength of 525 nm (SPECTRAmax Gemini XS, Molecular Devices).

### 4.5. HO-1 Activity

HO enzyme activity was measured as described previously [17]. Briefly, microsomes from harvested cells were added to a reaction mixture containing NADPH, rat liver cytosol as a source of biliverdin reductase, and the substrate hemin. The reaction was carried out for 1 h at 37 °C in the dark and terminated by the addition of 1 mL chloroform. The amount of extracted bilirubin in the sample was calculated using the difference in absorbance between 464 and 530 nm.

### 4.6. Preparation of Nuclear and Cytosolic Extraction

The cytosolic and nuclear fractions were obtained using NE-PER nuclear and cytoplasmic extraction reagents (Pierce Biotechnology, Rockford, IL, USA). Protein concentration was determined by the Bradford method (Bio-Rad, Irvine, CA, USA).

### 4.7. Western Blot Analysis

The cells were harvested on ice. Total cell lysates were prepared using lysis buffer (50 mM Tris, 150 mM NaCl, 5 mM EDTA, 1 mM DTT, 0.5% nonidet P-40, 100 mL phenylmethylsulfonylfluoride, 20 mM aprotinin, and 20 mM leupeptin, pH 8.0) and centrifugation at 15,000× *g* for 10 min. Protein concentration was determined by the Bradford method (Bio-Rad). Equal amounts of protein for each sample were resolved using sodium dodecyl sulfate-polyacrylamide gel electrophoresis (SDS-PAGE) and then transferred onto polyvinylidene fluoride (PVDF) membranes (Millipore, Cork, Ireland). The membranes were blocked with 5% skimmed milk and sequentially incubated with primary antibody and horseradish peroxidase-conjugated secondary antibody, followed by ECL detection (Amersham Pharmacia Biotech, Piscataway, NJ, USA).

### 4.8. Luciferase Assay

To construct the antioxidant response element (ARE)-luciferase vector, tandem repeats of double-stranded oligonucleotides spanning the Nrf2 binding site (5’-TGACTCAGCA-3’) were introduced into the restriction sites of the pGL2 promoter plasmid (Promega, Madison, WI, USA). All transfection experiments were performed using lipofectamine reagent (Invitrogen, Carlsbad, CA, USA) according to the manufacturer’s instructions. For luciferase assays, the cell lysate was first mixed with the luciferase substrate solution (Promega) and luciferase activity was measured using a luminometer. For each experiment, luciferase activity was determined in triplicate and normalized using β-galactosidase activity for each sample.

### 4.9. Statistical Analysis

All results are expressed as means ± S.D. at least three independent experiments. To compare three or more groups, one-way analysis of variance was performed followed by a Newman-Keuls *post-hoc* test. Statistical analysis was performed using GraphPad Prism software version 3.03 (GraphPad Software Inc., San Diego, CA, USA).

## 5. Conclusions

In conclusion, this study demonstrated that, BJ-1201, a 6-(diphenylamino)-2,4,5-trimethyl-pyridin-3-ol compound, reduced glutamate-induced cell cytotoxicity and ROS production in mouse hippocampal HT22 cells. Furthermore, we found that BJ-1201 also affected the expression of HO-1 through JNK or Nrf2 pathways, and it attenuated the inhibition of cell cytotoxicity or ROS production through HO-1 expression. These results suggest that BJ-1201 has the potential to reduce oxidative stress in neurodegenerative disease via the expression of HO-1. Thus, we will do the further study to confirm that is the specific mechanism of glutamate to induce oxidative via system Xc^−^ cysteine/glutamate exchanger or other glutamate receptors using antagonist of NMDA receptors.

## Figures and Tables

**Figure 1:** Effects of BJ-1201 on glutamate-induced oxidative neurotoxicity. (**a**) The structure of BJ-1201; (**b**) HT22 cells were incubated for 72 h with various concentration of BJ-1201; (**c**) HT22 cells were pre-treated with BJ-1201 for 12 h and then incubated for 12 h with glutamate (10 mM). Cell viability was measured by MTT assay; (**d**) Exposure of HT22 cells to glutamate increased ROS production. Each bar represents the mean ± S.D. of three independent experiments. * *p* < 0.05 compared with glutamate. Trolox (100 μM) was used as the positive control.

**Figure 2:** Effects of BJ-1201 on HO-1 expression in HT22 cell. (**a**) Cells were incubated for 18 h with sample (1–20 μM). Expression of HO-1 was determined by western blot analysis; (**b**) HO activity was determined via bilirubin formation at 12 h after treatment with various concentrations of BJ-1201. Each data represents the mean ± S.D. of three independent experiments are shown. CoPP (10 μM) was used as the positive control. * *p* < 0.05 compared with control group.

**Figure 3:** Effects of BJ-1201-induced MAPK activation in HT22 cells. Cells were treated with 20 μM BJ-1201 for the indicated times. Cell extracts were analyzed by western blot with antibodies specific for (**a**) phosphorylated ERK1/2 (p-ERK); (**b**) phosphorylated JNK (p-JNK); or (**c**) phosphorylated p38 (p-p38). Membranes were stripped and re-probed for the total form of each MAPK as a control, and representative blots of three independent experiments are shown. Each data represents the mean ± S.D. of three independent experiments are shown. * *p* < 0.05 compared with control group.

**Figure 4:** Effects of BJ-1201 on MAPK dependent HO-1 expression and cytoprotection in HT22 cells. (**a**) Cells were pretreated for 1 h with the specific inhibitor PD98059 (40 μM), SB203580 (20 μM), and SP600125 (25 μM), and then treated with 20 μM BJ-1201 for 18 h. Western blotting was then performed with HO-1 antibody; (**b**) Cells were treated with 20 μM BJ-1201 in the presence or absence of each specific inhibitors and SnPP (50 μM) for 12 h were exposed to 5 mM glutamate for 12 h. Data represent the mean ± S.D. of three independent experiments. * *p* < 0.05 compared with control group. ^#^ *p* < 0.05 compared with BJ-1201. ** *p* < 0.05 compared with glutamate (10 mM). ^$^ *p* < 0.05 compared with glutamate + BJ-1201.

**Figure 5:** Effects of BJ-1201 on Nrf2 nuclear translocation in HT22 cells. (**a**) Cells were treated with 30 μM BJ-1201 for 0.5, 1, and 1.5 h. Nrf2 protein was detected by western blot analysis; (**b**) Cells were transfected with ARE-luciferase of control vector were incubated for 1 h with the indicated concentrations of BJ-1201. Cells were assayed for luciferase activity as the fold induction by normalizing the transfection efficiency and dividing the values from each experimental sample relative to the control. Data represent the mean ± S.D. of three independent experiments. * *p* < 0.05 compared with control group.

## Abbreviations

The following abbreviations are used in this manuscript:

HO-1	heme oxygenase-1
Nrf2	nuclear transcription factor erythroid-2 related factor 2
AREs	antioxidant response elements
MAPKs	mitogen-activated protein kinases
